# The Performance of Artificial Intelligence Translation App in Japanese Language Education Guided by Deep Learning

**DOI:** 10.1155/2022/7962722

**Published:** 2022-05-18

**Authors:** Yi Wang

**Affiliations:** International School, Yunnan Minzu University, Kunming 650504, Yunnan, China

## Abstract

With recent technological advances in wireless networks and the Internet, social media has become a vital part of the daily lives of people. Social media like Twitter, Facebook, and Instagram have enabled people to instantly share their thoughts and ideas about a particular topic or person's life. Emotion classification in Twitter data remains a hot search topic in the field of artificial intelligence (AI). Though several models have been developed for tweet data in English, it is still needed to develop an effective tweet emotion classification for the Japanese language. In this aspect, this work develops a new artificial intelligence with an Optimal Long Short-Term Memory-Based Japanese Tweet Emotion Classification (OLSTM-JTCC) model in wireless networks. The proposed OLSTM-JTCC technique aims to examine emotions and categorises them into proper class labels. The proposed OLSTM-JTCC technique initially employs the TF-IFD model for the extraction of feature vectors. Besides, the OLSTM model is used to classify the tweet data into different types of emotions that exist within it. In order to improve the classification capability of the LSTM model, the Henry gas solubility optimization (HSGO) algorithm is applied as a hyperparameter optimizer. The performance validation of the OLSTM-JTCC technique took place using Japanese tweets, and the comparative results highlighted the better performance of the OLSTM-JTCC technique in terms of different measures.

## 1. Introduction

The teaching and translation of the Japanese language currently face new challenges and opportunities as a result of the rapid development of artificial intelligence technologies. Using a natural language processing ecosystem, people can enhance and personalise Japanese education. Japan's educational information technology will benefit from this, as will some of the existing issues. Impacting AI's advancement “Natural” languages such as Chinese, English, and Russian are some of the most widely spoken in the world [1]. Using computers, people are able to interpret and understand natural language and then put that knowledge to use. Text and speech, as well as the most common ways they are said, are all included in this category. Everything from grammar to semantics to pragmatics is covered [2]. The intended audience consists of intelligent individuals. Research in the social sciences, linguistics, and cognitive sciences is necessary if artificial intelligence is to develop a system that can process natural language [3]. With the development of breakthroughs in artificial intelligence and natural language processing, humans and computers can now converse in natural language. AI is being used by people in many areas of life at the moment. Using natural language processing, students in Japan can now converse in Japanese with computers and practise their language abilities through machine translation, voice navigation, intelligent robot dialogue, and composition corrections [4]. It is a difficult to implement AI and NLP in Japanese classrooms. It is not uncommon for students to come in all different sizes and shapes, as well as with a diverse spectrum of interests [5]. A student's previous knowledge of the Japanese language will determine which classes they should take [2]. It is possible for students' grammatical foundations and foreign language proficiency to alter the quality and efficacy of Japanese instruction. Artificial intelligence and natural language processing algorithms are unable to effectively translate literary images.

The lack of imagery in literary works may make it difficult to employ natural language processing algorithms to translate literary works [6]. A successful translation from one language to another is necessary for it to be a success. Additionally, it can represent the literary work and the author's objective in terms of language and style [7]. Language in nature contains a vast range of phrases and meanings because of its limited vocabulary and grammar. The lack of natural word segmentation in Japanese makes language processing more challenging than in other languages [8]. The computer's use of separators after each word causes semantic ambiguity in the Japanese translation, resulting in improper processing at all levels. Natural language processing can be difficult to execute because of the inherent ambiguity in linguistic units [9]. Artificial intelligence (AI) has a difficult time parsing cultural implications in human speech. Fluency in the country's native language is necessary for understanding its culture [10]. The oral tradition of language serves as a vehicle for the transmission of cultural heritage. The quality of Japanese education is being harmed by translations that are out of step with the modern context and culture due to artificial intelligence and natural language processing technology. Keep up with the pace of modern society by upgrading your artificial intelligence and natural language processing technologies on a regular basis [11]. Many new words and expressions have appeared to keep up with the rapid rise of the digital age, and as a result, our vocabulary continues to grow. Natural language processing now uses terms like “I'm too far south” and “Chuan Jianguo [12].” It is impossible to explain the meaning of these words unless you know their origins. In technology, intelligent interactivity is used to the greatest extent. A new language usually necessitates the combined efforts of the student and teacher. This is the only strategy that has been proven to be effective in increasing pupil comprehension. It is easier when there is a lot of information flowing in and out of it. The class as a whole is able to comprehend the language's core because each student has their own pronunciation and study technique [13]. Teachers are unable to evaluate the intellectual achievement of their students. It is possible that this will make it harder for students to tell one pupil from another. The use of existing artificial intelligence technologies to programme relevant data will benefit students immensely.

Teachers can, for example, make use of a system for processing human-computer dialogue [14]. When designing the system, keep in mind the wide range of learning styles represented by your pupils. Customizing the system's pages and the pronunciation options available will allow you to better suit the needs of your students. It is possible for a user to interact with a system by either typing or speaking to it. If the system is presented in an anthropomorphic way, students may be more attracted to studying Japanese. Students can now use the voice input device while reading long and complex Japanese sentences with the development of the addition of real-time voice interaction [15]. Using current technologies, it is now possible to analyse and identify errors in the Japanese language input. Student memory can be helped by generating hypothetical questions from the statements they just made, with the development of a computer programme that listens to their speech. Approaches like these help extroverts adapt more easily to the Japanese language and culture. With the interactive teaching method, introverted students and those with weak academic backgrounds will not be affected. With basic assertions, students can be taught on a case-by-case basis.

Natural language processing technology must be included in Japanese language instruction if it is to keep pace with the most current advances in artificial intelligence [16]. Teachers in the Tang dynasty may have utilised natural language processing to help students plan routes for Japanese experts who came to visit. Tang Dynasty wealth can be experienced through computer-mediated communications while students study about China and Japan's history, economy, culture, and society. As an additional stage in the educational process, courses in Japanese literature and cinema appreciation should be made available in schools for students to enhance their artistic abilities using natural language processing technologies. More and more students are using Japanese animation as a way of supplementing their education. In this way, teachers can fully utilise animation, film, and television while also allowing students to use the technology for dubbing and production, capturing students' attention, and stimulating their interest in natural language processing technology and ensuring that students are fully integrated into Japanese teaching classes at all levels of educational establishment. Science-based courses should be used to teach students how to analyse data [17]. When it comes to writing in Japanese, many students turn to translation software as a last resort. Students should be required to learn how to use translation software in the classroom. Interpreting techniques such as natural language processing should be taught to students as well. This should be a basic skill for all students. College students and young professionals may benefit from studying translation software and websites in depth. To get the greatest results from your translations, become an expert in debugging any software or websites that you use. To allow pupils to learn both Japanese and English, the Japanese education system should become multilingual. These include intelligent agents, natural language processing, and data mining. People are increasingly turning to these tools in order to expand their linguistic repertoire. Natural language processing was created by combining teaching principles with artificial intelligence. Language processing technologies can be used by schools to tackle educational challenges [18]. Because of the use of a teaching platform in an offline Japanese classroom, teachers can keep track of their students' development and make quick adjustments to their teaching methods. Students in Japan will benefit from this knowledge. Students can use the teaching platform's recommended content to augment their classroom Japanese learning. The use of artificial intelligence on the Internet can help with educational content, recommendations, and the detection of accomplishments. It is possible to generate student-specific learning files using students' voices, texts, and expressions. Many new technologies are being developed with the assistance of artificial intelligence and natural language processing (NLP) [19]. With more authority and time on their hands, people can improve Japanese public school education. Besides these limitations, this study used deep learning technique for evaluating Japanese translation apps.

## 2. Materials and Methods

In this work, a novel OLSTM-JTCC technique has been developed for the detection and classification of emotions in Japanese tweets. It mainly aims to investigate and categorise emotions into distinct classes. The proposed OLSTM-JTCC technique follows a three-stage process, namely, TF-IDF-based feature extraction, LSTM-based classification, and HSGO-based hyperparameter optimization. The detailed working of these processes is offered in the succeeding sections.

### 2.1. TF-IDF Vectorizer

The TF-IDF model is used for representing a term's relative importance in the record. The subsequent factor of the model is that term frequency (TF) is essential, which denotes the number of occurrences of a word in the dataset [1]. It can be defined as follows:

(1) $$\begin{array}{c} TF\left(t,d\right)=\frac{number\;of\;times\;t\;occurs\;in\;a\;do\;cument{\;}^{\prime }d{\;}^{\prime }}{total\;number\;of\;wor\;ds\;in\;do\;cument{\;}^{\prime }d{\;}^{\prime }}. \end{array}$$

Then, the inverse document frequency (IDF) can be used to represent how notable a term is in the whole dataset. The IDF can be formulated using the following:

(2) $$\begin{array}{c} IDF\left(t\right)=\;\log_{e}\left(\frac{\text{total number of documents}}{\text{number of documents with term t in it}}\right). \end{array}$$

Afterward, the TF-IDF can be defined, which is identical to the inverse document frequency combined with TF, as provided in the following:

(3) $$\begin{array}{c} TF‐IDF\;\left(t,d\right)=TF\left(t,d\right)*IDF\left(t\right). \end{array}$$

The TF‐IDF model extracts the features and highly relevant terms for emotion classification in Japanese tweets.

### 2.2. LSTM-Based Emotion Classification

During the emotion classification process, the LSTM model receives the feature vectors as input and determines the proper class labels. In general, the RNN network examines the input hidden series pattern through the concatenation of preceding data with present data from spatial and temporal dimensions and predicts the future classification. Even though RNN could extract the hidden time‐sequence pattern in consecutive information (that is, video, sensor, or audio data), it was incapable of remembering/holding longer data for a longer period and failed to handle the problem of having longer‐term sequence. This kind of issue is mentioned as vanishing or exploding gradients that overcomes a certain type of RNN called LSTM that has the ability to remember the data for a longer time [2]. The internal structure of LSTM comprises various gates (including output, input, and forget gate), whereby the gate processes the input from the prior gate and forwards them to the following gate thus controlling the data flow to the concluding output.  Figure 1 illustrates the framework of LSTM technique.

Each gate is generally managed through a sigmoid or tanh activation function, e.g., the input gate *i*_*t*_ is accountable for updating the data. The forget gate processes the input data from the input gate *i*_*t*_ also the state of preceding cell *C*_*t*−1_, as well eliminates the data from the existing state *C*_*t*_ while required where the output gate 0_*t*_ transmits the last output to the following LSTM unit and holds the output value for the following series calculation. Alternatively, recurrent unit *C*_*t*_ approximates the state of preceding cell *C*_*t*−1_ and existing input value *x*_*t*_ with tanh activation function where the value of *h*_*t*_ is estimated by the scalar product of 0_*t*_ and tanh of *C*_*t*_. Lastly, the final output is attained by passing *h*_*t*_ towards the softmax classification. Arithmetically the operation of abovementioned gate is formulated by

(4) $$\begin{array}{c} f_{t}=\Phi \left(\hat{W}\;.\left[h_{t-1^{\prime }}x_{t}\right]+B_{f}\right)\\ i_{t}=\Phi \left({\hat{W}}_{i}.\left[h_{t-1^{\prime }}x_{t}\right]+B_{i}\right)\\ C_{t}=\tanh\;\left({\hat{W}}_{C}.\left[h_{t-1},x_{t}\right]+B_{C}\right)\\ C_{t}=f_{t}xC_{t-1}+i_{t}xC_{t}\\ 0_{t}=\Phi \left(W_{0}\left[h_{t-1^{\prime }}x_{t}\right]+B_{0}\right)\\ h_{t}=o_{t}x\;\tanh\left(\Phi \left(C\right)\right.\\ \text{Output}=\text{softmax}\left(h_{t}\right). \end{array}$$

### 2.3. HSGO-Based Hyperparameter Tuning

In order to effectually adjust the hyperparameters such as batch size, learning rate, and epoch count, the HSGO algorithm has been employed to it. The HSGO algorithm is a recently developed metaheuristic methodology that simulates Henry's law [3]. Like the population‐based method, HGSO started by means of setting the early values for a group of *N* solutions (S) or gases as well as based on the searching area the equation can be expressed as follows:

(5) $$\begin{array}{c} X_{i}=Lb+\text{rand}*\left(Ub-Lb\right),\text{rand}\in \left[O,\;1\right], \end{array}$$

whereas *Lb* and *Ub* represent the lower and upper values in the searching space, correspondingly. The solution set *X* is clustered into equivalent amount of groups *N*_*g*_, and all the groups represent a kind of gas. All the groups have similar values for Henry's constant as follows:

(6) $$\begin{array}{c} H_{j}=l\times r_{1},\;j=1,2,\;N_{g},\;l=5E-2. \end{array}$$

Here, *l* indicates a constant and *r*_1_ denotes a random number. Next, define the optimal solution within all the groups. Next, the optimal solution over all the clustered groups can be defined. Afterward, Henry's coefficient (*H*_*j*_) for the *j*th group can be upgraded by

(7) $$\begin{array}{c} H_{j}\left(t+1\right)=H_{j}\left(t\right)\times \text{exp}\left(-C_{j}\times \left(\frac{1}{T\left(t\right)}-\frac{1}{T^{\theta }}\right)\right)\;,\;T\left(t\right)=\text{exp}\left(\frac{-t}{iter}\right), \end{array}$$

where *T*^*θ*^ and *iter* denote the temperature and constant values (set to 298.15), as well as the maximal value of iteration, correspondingly. The HGSO upgrades the solubility (*S*_*ij*_) of *X*_*j*_(*i*=1,2,  *N*) amongst each group:

(8) $$\begin{array}{c} S_{ij}\left(t\right)=K\times H_{j}\left(t+1\right)\times P_{ij}\left(t\right), \end{array}$$

whereas *K* represents a constant and *Pj*(*t*) denotes the partial pressure on *i*th gas with the *j*th cluster *j*:

(9) $$\begin{array}{c} P_{ij}\left(t\right)=l_{2}\times r_{1},\;j=1,2,\;N_{g},\;l_{2}=100. \end{array}$$

The solution *X*_*i*_ belonging to the *j*th cluster is upgraded as follows:

(10) $$\begin{array}{c} X_{ij}\left(t+1\right)=X_{ij}\left(t\right)+F_{g}\times r\times \eta \times \left(X_{ib}\left(t\right)-X_{ij}\left(t\right)\right)+F_{g}\times r\times \alpha \times \left(S_{ij}\left(t\right)\times X_{ib}\left(t\right)-X_{ij}\left(t\right)\right). \end{array}$$

whereas *η*=*β* × exp(−(*F*_*b*_(*t*)+*e*)/(*F*_*ij*_(*t*)+*e*)) describes the capacity of *i*th solution to communicate with other solutions in *j*th group. *F*_*b*_ signifies the optimal fitness value, and *F*_*ij*_ epitomizes the fitness value of *X*_*j*_ on *j*th group. *α* is the impact of solution on *X*_*j*_ of group*j*. *F*_*g*_ represent the flag value that changes the solution direction.

(11) $$\begin{array}{c} G_{ij}=G_{ij}^{\;\min}+r\times \left(G_{ij}^{\max}-G_{ij}^{\min}\right),\;i=1,2,\;N_{w},\\ N_{w}=N\times r\times \left(c_{2}-c_{1}\right)+c_{1},c_{1}=0.1,\text{ and}c_{2}=0.2. \end{array}$$

*G*_*ij*_ characterizes the solution *X*_*i*_ in *j*th group belonging to the worst solution.

## 3. Results and Discussion

Here, the performance of the OLSTM-JTCC model on the emotion classification of Japanese tweets is investigated.  Table 1 and Figure 2 provide the classification result analysis of the OLSTM-JTCC model under two emotion classes, namely, Joy and Sadness. The results display that the OLSTM-JTCC model has resulted in increased classifier results on both classes. In addition, the OLSTM-JTCC technique has identified the tweet as joy emotion with the *prec*_*n*_ of 98.14%, *reca*_*l*_ of 98.6%, and *F*_score_ of 98.28%.

Moreover, the OLSTM-JTCC model has recognized the tweet as sadness emotion with the *prec*_*n*_ of 98.64%, *reca*_*l*_ of 98.64%, and *F*_score_ of 98.47%.

Table 2 provides a comprehensive classification result analysis of the OLSTM-JTCC model with existing techniques.  Figure 3 provides a detailed precision, recall, and F-score analysis of the OLSTM-JTCC technique with other models. The figure exposes that the TF-IDF1 approach has resulted in lesser precision, recall, and F-score of 85.60%, 85.60%, and 85.60%.

Followed by, the TF-IDF3 model has obtained somewhat maximum precision, recall, and F-score of 90.20%, 90.20%, and 90.20%. Followed by, the BERT-FT technique has accomplished reasonable precision, recall, and F-score of 98.20%, 98.20%, and 98.20%. At last, the OLSTM-JTCC model has reached maximum precision, recall, and F-score of 98.39%, 98.62%, and 98.38%.

Figure 4 offers a brief accuracy analysis of the OLSTM-JTCC system with other models. The figure reports that the TF-IDF1 model has resulted in lower accuracy of 85.70%. Followed by, the TF-IDF3 model has obtained slightly increased accuracy of 90.10%. Along with that the BERT-FT technique has accomplished reasonable accuracy of 98.10%. However, the OLSTM-JTCC model has obtained improved accuracy of 98.54%.

By observing the abovementioned results, it is concluded that the OLSTM-JTCC model has effectually identified the emotions that exist in the Japanese tweets. In general, teachers in an offline Japanese classroom can monitor their students' progress and make quick adjustments to their teaching methods thanks to the use of a teaching platform. Use the teaching platform's recommended content to supplement classroom Japanese studies. Artificial intelligence (AI) on the Internet can help with educational content, recommendations, and the detection of accomplishments of students. Students' voices, texts, and expressions can be used to create student-specific learning files.

## 4. Conclusions

Social media has become an essential part of people's daily lives as a result of recent technological advancements in wireless networks and the Internet. Individuals can now express themselves about a particular subject or person's life in real time using social media platforms such as Twitter, Facebook, Instagram, and many others. Classification of emotions in Twitter data is still a popular AI research topic (AI). There are several models for tweet data in English, but it is still necessary to develop an effective classification system for the Japanese language. In this regard, this work develops a new artificial intelligence in wireless networks with an OLSTM-JTCC model for optimal long short-term memory-based Japanese tweet emotion classification. Using the proposed OLSTM-JTCC method, researchers hope to identify and classify emotions. Initial feature extraction is carried out using the TF-IFD model, which is used in the OLSTM-JTCC technique. OLSTM models are also used to categorise the tweet data into a variety of different emotional states. The Henry gas solubility optimization (HSGO) algorithm is used as a hyperparameter optimizer to improve the classification capability of the LSTM model. The OLSTM-JTCC technique was tested using Japanese tweets, and the comparison results showed that the OLSTM-JTCC technique performed better in terms of a variety of metrics.

## Figures and Tables

**Figure 1:** Structure of the LSTM model.

**Figure 2:** Result analysis of OLSTM-JTCC technique.

**Figure 3:** Comparative analysis of OLSTM-JTCC technique.

**Figure 4:** Accuracy analysis of OLSTM-JTCC technique with recent approaches.

**Table 1:** Result analysis of OLSTM-JTCC technique under two classes.

Class label	Precision	Recall	F-score
Joy	98.14	98.6	98.28
Sadness	98.64	98.64	98.47

**Table 2:** Comparative analysis of OLSTM-JTCC technique with recent approaches.

Methods	Precision	Recall	Accuracy	F-score
TF-IDF1	85.60	85.60	85.70	85.60
TF-IDF3	90.20	90.20	90.10	90.20
BERT-FT	98.20	98.20	98.10	98.20
OLSTM-JTCC	98.39	98.62	98.54	98.38

## Data Availability

The data used to support the ﬁndings of this study are available from the corresponding author upon request.
